# Continuous Psychological Nursing Based on Grey Clustering Algorithm in Patients after Transurethral Resection of Prostate

**DOI:** 10.1155/2022/5400479

**Published:** 2022-07-28

**Authors:** Peiting Lu, Cuiyun Wu

**Affiliations:** ^1^Urology Surgery, The Third People's Hospital of Hefei, Hefei, Anhui 230022, China; ^2^Nursing Department, The Third People's Hospital of Hefei, Hefei, Anhui 230022, China

## Abstract

**Objective:**

To explore the effect of continuous psychological nursing based on the grey clustering algorithm on erectile function, bad psychological emotion, and complications in patients after transurethral resection of prostate (TURP).

**Methods:**

98 patients who underwent TURP were randomly divided into observation and control groups (routine nursing). The observation group first used the grey clustering algorithm to evaluate the psychological intelligence, found patients with abnormal psychological behavior, and then implemented continuous psychological nursing combined with pelvic floor muscle exercise. The patients were followed up for 4 months. The International Index of Erectile Function-5 (IIEF-5), the incidence of complications, the Hamilton Depression Scale (HAMD), the Hamilton Anxiety Scale (HAMA) scores, and the nursing satisfaction were analyzed and compared between these two groups.

**Results:**

The grey clustering algorithm can accurately reflect the characteristics of patients' psychological changes. After targeted nursing, compared with the control group, the IIEF-5 in the observation group was higher [(24.87 ± 1.85) vs. (22.24 ± 1.47), *P* < 0.05], the incidence of total complications was lower (10.20% vs. 26.53%, *P* < 0.05), the score of HAMA was lower [(6.11 ± 2.57) vs. (10.98 ± 2.29), *P* < 0.05], the score of HAMD was lower [(6.97 ± 2.85) vs. (11.35 ± 2.19), *P* < 0.05], and the nursing satisfaction was higher (100% vs. 85.71%, *P* < 0.05).

**Conclusion:**

Mental intelligence evaluation based on the grey clustering algorithm combined with pelvic floor muscle exercise can significantly improve the rehabilitation effect of erectile function in patients after TURP, reduce the incidence of postoperative complications, and alleviate patients' anxiety and depression.

## 1. Introduction

Benign prostatic hyperplasia (BPH) is one of the common diseases in the male urinary system. Its primary clinical symptoms are urinary storage symptoms: frequent micturition, urgent micturition, and micturition symptoms (delayed initial micturition time, intermittent micturition, etc.) [1]. At present, patients with mild benign prostatic hyperplasia are mainly treated conservatively with drugs [2]. Moderate and severe patients are often accompanied by erectile dysfunction [3]. Surgical treatment is a commonly used program but easily leads to complications such as urinary tract infection, urinary retention, and urinary incontinence [4].

Patients undergoing prostatectomy are affected by many subjective and objective risk factors. They are prone to negative psychological emotions such as sleep disorder, anxiety, and depression [5], which will interfere with the rehabilitation of patients' erectile function [6]. How to treat erectile dysfunction and bad psychological emotion after benign prostatic hyperplasia is essential clinical research. Relevant studies have pointed out that men can effectively restore pelvic floor muscle tension and improve erectile dysfunction by using pelvic floor muscle functional exercise to repair pelvic floor muscle damage [7–9]. However, patients will have different abnormal psychology after the operation and reject pelvic floor functional exercise. Or it is difficult to persist for a long time [10]. At present, the psychological evaluation of patients after prostatectomy is still relatively simple, which is difficult to describe the psychological status of patients accurately [11].

As a mathematical method to solve the system of missing information, the grey clustering algorithm integrates automatic control and operational research methods, which can solve the grey problem in psychological evaluation [12]. This method has been applied to students' psychological evaluation and achieved ideal application results [13, 14]. This study attempts to use the grey clustering algorithm in the psychological assessment of patients after prostatectomy, and then implement more accurate nursing and pelvic floor functional exercises according to the evaluation results.

## 2. Data and Methods

### 2.1. Basic Data

From January 2018 to October 2020, 98 patients with benign prostatic hyperplasia planned to undergo transurethral resection of the prostate (TURP) in the Hefei Third People's Hospital. They were randomly divided into two groups: 49 cases in the observation group, with an average age of 72.15 ± 7.23 years, and 49 cases in the control group, with an average age of 73.81 ± 4.59 years. There was no significant difference in age, educational level, economic income, prostate volume, International Prostate Symptom Score (IPSS), IIEF-5, maximum urinary flow rate (Qmax), and residual urine (PVR) between the two groups (Table 1, *P* > 0.05). Before this study's implementation, it was reported to the hospital medical ethics committee for review and consent, and all patients signed the informed consent form.

### 2.2. Inclusion and Exclusion Criteria

Inclusion criteria are as follows: (1) the patients met the diagnostic criteria of the BPH international scoring scale, had the indication of prostatectomy, and were willing to undergo prostatectomy; (2) the patient's previous medication and treatment did not affect sexual function; (3) all patients signed informed consent.

Exclusion criteria are as follows: (1) widowers without wives; (2) patients with poor marital relationships; (3) patients with mental disorders; (4) patients with previous erectile dysfunction; (5) previous history of prostate surgery.

### 2.3. Nursing Methods

Patients in the control group were given routine nursing during hospitalization, including preoperative health education, postoperative monitoring of patients' vital signs, and exercise of bladder function. When the patients discharged from the hospital, routine oral education was carried out, the telephone contact card was distributed, the patients were instructed to follow up once a month, and the corresponding questionnaire and self-assessment scale were completed without out-of-hospital nursing intervention.

The patients in the observation group first used the grey clustering algorithm to evaluate their psychological intelligence. Those patients with abnormal psychological behavior implemented continuous psychological nursing and pelvic floor muscle training based on the control group.

#### 2.3.1. Establish a Continuous Psychological Nursing Group

The head nurse acts as the team leader, responsible for managing the content and plan and formulating rehabilitation materials and questionnaires. The members include 2 senior urologists and 5 nurses with more than 5 years of specialized nursing experience. All nurses are familiar with the continuous psychological nursing guidance procedures of TURP and related complications. All the members have received unified training. Each nurse is responsible for about 10 patients, and each has his responsibility. They carry out continuous psychological nursing for discharged patients according to the nursing plan. Doctors are responsible for answering questions and solving doubts about urinary diseases. All patients in the study group and their wives were pulled into the WeChat group when they were discharged from the hospital.

#### 2.3.2. Develop Patient Information Files

Include the patient's name, age, address, telephone, WeChat, diet, sleep, psychological status, urination, stool, medication at discharge, complications, and other information.

#### 2.3.3. WeChat Group Follow-up

On WeChat group, answer questions from 18 : 00 to 20 : 00 every Saturday, and answer questions at any time in case of emergency. Follow up with all patients through the WeChat group each month's first week. At the same time, give continuous psychological nursing guidance and pelvic floor muscle exercise guidance to patients, summarize and evaluate the continuous nursing situation of patients at the end of each month, and report to the head nurse. The follow-up time was 4 months after operation.

#### 2.3.4. Dietary Guidance

Ask patients about their diet on WeChat every month. It is suggested that the patients should eat more high-quality protein (such as chicken, fish, lean meat, and eggs), eat fat appropriately, and supplement a variety of vitamins and trace elements (such as shrimp, seafood, and leek).

#### 2.3.5. Family Nursing

The mental support of the patient's wife helps alleviate the patient's anxiety, depression, and other psychology, to promote the patient's early recovery. Therefore, the WeChat group did an excellent job in the ideological work of the patient's wife; asked him to communicate more with the patient, provide emotional comfort and care, take care and help in life, and help the patient get out of the shadow of the disease as soon as possible.

#### 2.3.6. Sexual Life Guidance

Two months after the operation, the patients were suggested that they could try sex life through the WeChat group. The nurse explained the operation changes to the patients and their spouses through WeChat video and told the patients that the occasional unsuccessful one-time life was not a permanent erectile dysfunction. Before and during sexual intercourse, both husband and wife must maintain a friendly and harmonious atmosphere and mood. They should care for each other and give their best, enhancing love and pleasure. Choose a warm, stable, and comfortable sexual intercourse environment.

#### 2.3.7. Guidance on Complication Prevention

In the first week of each month after discharge, the responsible nurse uses the WeChat group to explain in detail the possible complications of patients after discharge, find them in time, intervene, and prevent them. Patients with perineal skin exposed in urine will produce erythema, ulcer, and other perineal dermatitis. To keep the perineum clean, do an excellent job in skin care, select the correct cleaning solution, and reasonably use external medication.

#### 2.3.8. Adverse Psychological Intervention

Ask the husband and wife to cooperate. The wife should encourage her husband to find a favorable and quiet sexual life environment. Do not be impatient. Make full use of foreplay. If necessary, ask a psychologist for treatment. Be sure to enhance self-confidence and eliminate negative emotions such as tension, depression, and anxiety.

#### 2.3.9. Pelvic Floor Muscle Exercise

At admission, the responsible nurse instructed the patient to start pelvic floor muscle exercise 3 days before the operation and informed the patient of the importance and necessity of exercise. The patient lies on his side on the treatment bed. The responsible nurse wears disposable latex gloves, and the index finger is coated with paraffin oil, massages around the anus for a few seconds. When the anal sphincter is relaxed, slowly insert into the patient's anus and instruct him to tighten and relax the anus, just like a deliberate pause during defecation and urination. Keep the muscles tightened for 3-20 seconds each time, and then relax for 15 minutes each time.

Before the operation, the pelvic floor muscle exercises three times a day and can repeatedly practice each time. The exercise was suspended within 3 days after operation. 4-7 days after operation, exercise for about 8 minutes each time, three times a day, and adjust it in time according to the patient's main complaints of discomfort such as urethral tingling. After 7 days, pelvic floor muscle exercise is as before operation but should also pay attention to the patient's discomfort until 4 months after operation.

When exercising for the first time, the nurse will guide in person, and the rest will follow the doctor's advice and take the initiative to exercise. The responsible nurse conducted an international questionnaire survey on erectile function and adjusted the exercise time and times according to the results.

### 2.4. Psychological Evaluation Process

The grey clustering algorithm is used to evaluate the psychological state of patients after prostatectomy, as shown in Figure 1. According to the common psychological characteristics of patients after prostatectomy, construct the psychological intelligence evaluation index system, quantify the specific score of each index, collect the relevant data of each index, construct the evaluation, use the constructed model to evaluate the mental health level of patients, and obtain the evaluation results.

There are certain constraints on human cognitive ability, which cannot fully recognize the information describing the operation behavior of the system. As a result, in the process of actual human cognition, only the value range of relevant system parameters can be analyzed. The grey number can describe the number that can only understand the value range and cannot determine the specific value. In practical application, grey numbers can represent uncertain numbers in any interval or number set. Under the condition of obtaining partial distribution information, the tendency of the grey level to each number within its value range can be expressed by the whitening weight function. According to the difference of mental health of patients after prostatectomy, their mental state indexes are divided into three grey categories: good, ordinary, and morbid.  Figure 2 shows the different indicators of patients' psychology.

The grey evaluation based on the trigonometric whitening weight function of calculation points is used to construct the psychological state of patients. The specific process is as follows.

1. Determine the geometric midpoint between [A1, A2], [A2, A3], and [A3, A4] of each row of indicators in the grey number classification table of patients' mental health evaluation indicators:

(1) $$\begin{array}{c} \gamma_{k}=\frac{\left(a_{k}+a_{k+1}\right)}{2},k=1,2,3. \end{array}$$

(2) Let the *f*( ) value of *r*_*k*_ belonging to the *k* grey class be 1, and construct the geometric centers of *k* − 1 and *k* + 1 as the *r*_*k*−1_ and *r*_*k*+1_. The observed value of an index in the evaluation index system is represented by *x*, and the membership ∫_*j*_^*k*^(*x*) belonging to grey class *k* is determined by

(2) $$\begin{array}{c} f_{j}^{k}\left(x\right)=\left\{\begin{array}{cc} 0, & x∄\left[r_{k-1},r_{k+1}\right]\\ \frac{x-r_{k-1}}{r_{k}-r_{k-1}}, & x\in \left[r_{k-1},r_{k}\right]\\ \frac{x-r_{k+1}-x}{r_{k+1}-r_{k}}, & x\in \left[r_{k},r_{k+1}\right] \end{array}\right\}. \end{array}$$

(3) The weight *Z*_*j*_ of the jth evaluation index in the process of comprehensive clustering is calculated according to the proportion of the total score of each index value in the overall score of the evaluation index system. The calculation formula is as follows:

(3) $$\begin{array}{c} Z_{j}=\frac{E_{j}}{\text{Total}}, \end{array}$$

where *E*_*j*_ and Total are the total score of the *j*th evaluation index and the overall score of the index system, respectively.

(4) *x*_*ij*_ represents the observed value of the ith patients' mental health evaluation index *j*. *x*_*ij*_  is introduced into the corresponding membership degree ∫_*j*_^*k*^ (*x*) to determine the comprehensive clustering coefficient of patient *i* on grey class *K∂*_*j*_^*k*^. Determine the grey class *k*^∗^ of patient *i* by using

(4) $$\begin{array}{c} 1\leq \dddot{k}\leq 3\left(\partial_{j}^{k}\right)=\partial_{j}^{k^{*}}. \end{array}$$

### 2.5. Observation Indicators

1. International questionnaire on erectile function 5 (IIEF-5): IIEF-5 scores of patients in the two groups were investigated on the first day before nursing and the fourth month after nursing. The questionnaire was completed through direct delivery to patients or WeChat. If the total score is less than 22, it is ed, and if the total score is more than 22, it is normal (Cronbach′s *α* = 0.85). IIEF-5 score is directly proportional to erectile function
2. The incidence of complications was compared between the two groups
3. Evaluation of psychological status: the results of HAMA (Cronbach′s *α* = 0.90) and HAMD (Cronbach′s *α* = 0.88) were tested on the first day before nursing and the fourth month after nursing through direct delivery to patients or WeChat. HAMA ≥7 points have anxiety, and <7 points have no anxiety. HAMD ≥7 points have depression, and <7 points have no depression
4. Nursing satisfaction: the self-designed satisfaction questionnaire was adopted, and the total score was 100 points. The questionnaire was completed through direct delivery to patients or WeChat. Satisfaction = (very satisfied + satisfied)/total × 100%. Score ≥90 points is very satisfied; 60-90 points are satisfactory; <60 is not satisfied

### 2.6. Statistical Methods

SPSS 20.0 statistical software was used for data analysis. The measurement data were in line with the normal distribution and expressed in (*x* ± *s*). The differences between measurement data groups were compared by independent sample *t*-test and one-way ANOVA, and the counting data were analyzed by *χ*^2^ and Fisher exact probability test. The difference was statistically significant (*P* < 0.05).

## 3. Results

### 3.1. Mental Health Evaluation Results

Figure 3 shows the weight calculation results of each evaluation index in this method's evaluation index system, obtained according to the proportion of the score in the overall score of the evaluation index system. According to the quantitative value of each index, the overall score of each application object is obtained (Figure 4). It can be seen that the scores of patients can be roughly divided into two categories. One category with a score of more than 100 points is classified as morbid grey, and the other category with a score of less than 100 points is classified as ordinary grey.

Through the intelligent mental health evaluation, we can understand the current mental health level and main problems of patients and conduct psychological counseling and related treatment according to the evaluation results. After the treatment period, we use this method to conduct mental health evaluation again. It is found that the mental health level of all patients has been significantly improved, and the improvement of morbid grey-scale patients is more obvious (Figure 5).

### 3.2. Comparison of IIEF-5

Before nursing, there was no statistical difference of IIEF-5 between the two groups. After nursing, IIEF-5 (24.87 ± 1.85) in the observation group was higher than that in the control group (22.24 ± 1.47) (*P* < 0.05). The detail is shown in Table 2.

### 3.3. Comparison of Incidence of Complications

The total complications in the observation group (10.20%) were lower than those in the control group (26.53%) (*x*^2^ = 4.356, *P* = 0.037); in the observation group, the complications were urinary incontinence (2, 4.08%), urinary system infection (1, 2.04%), urinary retention (1, 2.04%), and urethral bleeding (1, 2.04%). In the control group, those and other complications were 10.20%, 4.08%, 4.08%, 6.12%, and 2.04%, respectively.

### 3.4. Comparison of Psychological Condition

Before nursing, there was no statistical difference of HAMA and HAMD between the two groups. After nursing, the score of HAMA in observation group was lower [(6.11 ± 2.57) vs. (10.98 ± 2.29), *P* < 0.05], and the score of HAMD was lower [(6.97 ± 2.85) vs. (11.35 ± 2.19), *P* < 0.05]. The detail is shown in Table 3.

### 3.5. Comparison of Nursing Satisfaction

The satisfaction of 49 patients in the observation group (continuous psychological nursing combined with pelvic floor muscle exercise) was 100% (49/49), which was significantly higher than 85.71% (42/49) in the control group (*P* < 0.05). The detail is shown in Table 4.

## 4. Discussion

Benign prostatic hyperplasia is noncancerous hyperplasia of the prostate. The cause of this disease is related to the change of male androgen, and there may be no obvious symptoms in the early stage. After the age of 45, the male prostate has hypertrophy and hyperplasia with different stages, and the incidence rate increases rapidly [15]. In the course of illness, a considerable number of patients have different degrees of erectile dysfunction, so patients suffer from unprecedented physiological and psychological pressure [16], which interferes with the quality of work and life. The causes of benign prostatic hyperplasia and erectile dysfunction can be divided into two categories: organic factors and psychological factors [17]. The main organic factors are the sympathetic nerves of the genitourinary system dominating the bladder and prostate and the penile autonomic plexus controlling penile erection, which are homologous to the pelvic plexus. Due to the origin of the same plexus, the patient's prostate gradually proliferates and hypertrophies, and the excitability of negative feedback sympathetic nerve increases daily [18]. Then, the excitability of penile autonomic plexus controlling penile erection also increases daily, which leads to difficulty in penile erection function [19], and the corresponding homologous nerve controlling erectile function may be burned during electrotomy. The main mental and psychological factors are the patient's excessive pressure, anxiety, and depression, followed by the increase of sympathetic nerve excitability in the body and the functional contraction of penile cavernous smooth muscle, resulting in ED. During illness and after surgery, sexual intercourse is not successful occasionally, resulting in great psychological obstacles and a very tense state in each sexual life, lack of sexual knowledge, mistakenly believe that sexual intercourse cannot be performed after surgery, fear that sexual intercourse will aggravate the disease, worry about gain and loss, or improper or insufficient sexual stimulation. In addition to aiming at the cause of erectile dysfunction, correcting bad lifestyle, treating basic diseases, and properly using phosphodiesterase 5 inhibitors, erectile dysfunction depends on psychological counseling and functional exercise measures. With social progress, people's material living standards are improving day by day, and they are more concerned about the quality of life, which needs to be improved day by day. Therefore, the implementation of continuous psychological nursing combined with pelvic floor muscle exercise to improve erectile dysfunction is a great progress in nursing [20].

Continuous nursing has been widely used in recent years. It usually refers to the seamless care provided from the hospital to the family according to the patient's condition needs, including the discharge doctor's order guidance formulated by the hospital and the patient's regular follow-up at home and out-of-hospital physical and psychological rehabilitation nursing counseling [21]. The continuous nursing we adopted this time is mainly psychological nursing counseling, supplemented by other nursing, so it is named continuous psychological nursing. WeChat official account is a one-to-one and one-to-many media sexual activity, which plays an important role in the health guidance of continuous psychological nursing. Pelvic floor muscle exercise is also called Kegel exercise, often called anal lifting exercise. It can treat diseases such as uterine prolapse, female sexual dysfunction, and urinary incontinence [22–24]. The cavernous nerve controlling male penile erection and the sympathetic and parasympathetic nerves innervating prostate and bladder all come from pelvic plexus. Because of neural homology, exercising pelvic floor muscles can improve pelvic plexus's innervation ability, improving patients' erectile function and reducing the incidence of ed. However, we also need to see that continuous nursing costs are very high and the nursing knowledge is not targeted. After evaluating patients' mental health through grey clustering algorithm, patients' health problems can be found timely and accurately, to implement a more purposeful nursing plan. This study found that after nursing, IIEF-5 (24.87 ± 1.85) in the observation group was higher than that in the control group (22.24 ± 1.47) (*P* < 0.05). Therefore, the researchers' application of psychological counseling and pelvic floor muscle exercise can improve the curative effect of treating sexual dysfunction; the above counter evidence shows that erectile dysfunction after benign prostatic hyperplasia should be diagnosed in time, treated early, and intervened by psychological nursing first; otherwise, it may leave sequelae.

Continuous psychological nursing, through out-of-hospital follow-up, functional exercise guidance, and a series of physical, mental, and psychological nursing suggestions for discharged patients, cultivates good self-care ability and self-management skills; promotes the early physical and mental recovery of patients; improves the quality of life of patients; strengthens the relationship between nurses, doctors, and patients; intervenes the bad psychological emotions of patients; gives full play to the subjective initiative of patients; and creates a peaceful and harmonious society. After prostatectomy, the excitability of the penis is reduced, and the sympathetic function is reduced; it is responsible for the cause of erectile dysfunction and can promote the homologous muscle circulation of the pelvic floor. It can enhance the muscle function related to the erectile dysfunction. This continuous psychological nursing combined with pelvic floor muscle exercise is mainly tailored to the two causes of erectile dysfunction. Dietary guidance provides patients with a healthy and strong body; pelvic floor muscle exercise corrects the organic factors of erectile dysfunction; sexual life guidance and adverse psychological intervention completely solved the mental and psychological factors of patients, such as tension, anxiety, and depression; family friendly nursing enables patients to obtain spiritual and material support from their wives, encourages patients to eliminate psychological obstacles, often participate in social activities, and avoid mental and psychological diseases. Therefore, wife support is an irreplaceable intervention behavior in the treatment and rehabilitation of patients with sexual dysfunction [25], so the patients with poor husband wife relationship are excluded. The total complication rate in the continuous psychological nursing combined with pelvic floor muscle exercise group was 10.20%, which was significantly lower than 26.53% in the control group (*P* < 0.05). However, the incidence of single complications such as urinary incontinence, urinary system infection, and urinary retention is not statistically significant compared with the control group, which may be related to the fewer cases enrolled this time. It is hoped that the follow-up study will increase the cooperation of multiple departments and centers.

In fact, not all patients have psychological problems. Using the same intervention scheme for all patients not only wastes data, but also may cause the scheme of some patients. The patients in the observation group first used the grey clustering algorithm to evaluate the psychological intelligence and found that the patients with abnormal psychological behavior implemented continuous psychological nursing and pelvic floor muscle training. Eliminating the patient's psychological disorder will improve his sexual life. In this study, the HAMA and HAMD scores of the two groups of patients on the first day before nursing were relatively high, indicating that physical diseases can aggravate or induce depression, anxiety, and psychological diseases, especially urinary diseases and especially male diseases. Therefore, after 4 months of targeted continuous psychological nursing, the HAMA and HAMD scores of the observation group were significantly lower than those of the control group (*P* < 0.05). It shows that continuous psychological nursing can reduce the psychological and physiological pain of patients and improve the quality of life. With the elimination of patients' sexual dysfunction and the gradual establishment of positive and progressive mentality, patients' anxiety and depression gradually disappeared, which showed that the patients in the observation group benefited a lot from their daily life and work. Accordingly, the nursing satisfaction was 100%, significantly higher than 85.71% in the control group, and the difference was statistically significant.

## 5. Conclusion

In summary, the mental intelligence evaluation based on the grey clustering algorithm combined with pelvic floor muscle exercise can significantly improve the rehabilitation effect of erectile function in patients after TURP, reduce the incidence of postoperative complications, and alleviate patients' anxiety and depression.

## Figures and Tables

**Figure 1:** Psychological evaluation process in patients with TURP.

**Figure 2:** Different indicators of patients' psychology in patients with TURP.

**Figure 3:** Calculation of weight index.

**Figure 4:** Distribution of psychological evaluation scores.

**Figure 5:** Calculation results of quadratic comprehensive clustering coefficient (all *P* < 0.001).

**Table 1:** Comparison of clinical data between the two groups.

Clinical features	Observation group (*n* = 49)	Control group (*n* = 49)	*t*/*X*^2^	*P*
Age(year)	72.15 ± 7.23	73.81 ± 4.59	0.817	0.416
Education			0.042	0.838
Bachelor's degree or above	29	28		
Junior college or below	20	21		
Family economic income			0.041	0.839
<8 (10000/year)	27	28		
≥8 (10000/year)	22	21		
Prostate volume (ml)	65.25 ± 3.62	63.79 ± 1.23	2.008	0.056
IPSS (score)	21.35 ± 2.95	22.42 ± 3.16	3.254	0.956
PVR (ml)	63.85 ± 35.29	61.96 ± 40.47	2.102	0.785
Qmax (ml/min)	6.75 ± 1.35	7.25 ± 2.56	3.251	1.024
IIEF-5	14.95 ± 3.21	15.08 ± 2.56	0.058	0.943

**Table 2:** Comparison of IIEF-5 between the two groups.

Group	Before nursing	After nursing
Observation group	20.75 ± 2.65	24.87 ± 1.85
Control group	20.23 ± 3.85	22.24 ± 1.47
*F*	0.314	19.063
*P*	0.577	0.000

**Table 3:** Comparison of psychological status between the two groups.

Group	HAMA	HAMD
Observation group		
Before nursing	14.38 ± 1.19	17.15 ± 2.04
After nursing	6.11 ± 2.57	6.97 ± 2.85
*t*	5.451	3.652
*P*	0.006	0.027
Control group		
Before nursing	14.85 ± 1.58	16.97 ± 1.46
After nursing	10.98 ± 2.29	11.35 ± 2.19
*t*	4.652	2.852
*P*	0.014	0.046

**Table 4:** Comparison of nursing job satisfaction between the two groups.

Group	*n*	High	Normal	Dissatisfied	Satisfaction
Observation group	49	29	20	0	100%
Control group	49	25	17	7	85.71%
*x* ^2^	5.538				
*P*	0.019				

## Data Availability

The data used to support the findings of this study are available from the corresponding author upon request.
